# Therapeutic effect of nanoliposomal PCSK9 vaccine in a mouse model of atherosclerosis

This article has been retracted.

**DOI:** 10.1186/s12916-019-1457-8

**Published:** 2019-12-10

**Authors:** Amir Abbas Momtazi-Borojeni, Mahmoud Reza Jaafari, Ali Badiee, Maciej Banach, Amirhossein Sahebkar

**Affiliations:** 1 Nanotechnology Research Center, Bu-Ali Research Institute, Mashhad University of Medical Sciences, Mashhad, Iran; 2 Department of Medical Biotechnology, Student Research Committee, Faculty of Medicine, Mashhad University of Medical Sciences, Mashhad, Iran; 3 Nanotechnology Research Center, Pharmaceutical Technology Institute, Mashhad University of Medical Sciences, Mashhad, Iran; 4 Biotechnology Research Center, Pharmaceutical Technology Institute, Mashhad University of Medical Sciences, Mashhad, Iran; 5 Department of Pharmaceutical Nanotechnology, School of Pharmacy, Mashhad University of Medical Sciences, Mashhad, Iran; 6 Department of Hypertension, WAM University Hospital in Lodz, Medical University of Lodz, Zeromskiego 113, Lodz, Poland; 7 Polish Mother’s Memorial Hospital Research Institute (PMMHRI), Lodz, Poland; 8 Neurogenic Inflammation Research Center, Mashhad University of Medical Sciences, Mashhad, Iran; 9 School of Pharmacy, Mashhad University of Medical Sciences, Mashhad, Iran

**Keywords:** Atherosclerosis, Low-density lipoprotein cholesterol, PCSK9, Immunotherapy

## Abstract

**Background:**

Proprotein convertase subtilisin/kexin 9 (PCSK9) is an important regulator of low-density lipoprotein receptor (LDLR) and plasma levels of LDL cholesterol (LDL-C). PCSK9 inhibition is an efficient therapeutic approach for the treatment of dyslipidemia. We tested the therapeutic effect of a PCSK9 vaccine on dyslipidemia and atherosclerosis.

**Methods:**

Lipid film hydration method was used to prepare negatively charged nanoliposomes as a vaccine delivery system. An immunogenic peptide called immunogenic fused PCSK9-tetanus (IFPT) was incorporated on the surface of nanoliposomes using DSPE-PEG-maleimide lipid (L-IFPT) and adsorbed to Alhydrogel® (L-IFPTA^+^). The prepared vaccine formulation (L-IFPTA^+^) and empty liposomes (negative control) were inoculated four times with bi-weekly intervals in C57BL/6 mice on the background of a severe atherogenic diet and poloxamer 407 (thrice weekly) injection. Antibody titers were evaluated 2 weeks after each vaccination and at the end of the study in vaccinated mice. Effects of anti-PCSK9 vaccination on plasma concentrations of PCSK9 and its interaction with LDLR were determined using ELISA. To evaluate the inflammatory response, interferon-gamma (IFN-γ)- and interleukin (IL)-10-producing splenic cells were assayed using ELISpot analysis.

**Results:**

L-IFPTA^+^ vaccine induced a high IgG antibody response against PCSK9 peptide in the vaccinated hypercholesterolemic mice. L-IFPTA^+^-induced antibodies specifically targeted PCSK9 and decreased its plasma consecration by up to 58.5% (− 164.7 ± 9.6 ng/mL, *p =* 0.0001) compared with the control. PCSK9-LDLR binding assay showed that generated antibodies could inhibit PCSK9-LDLR interaction. The L-IFPTA^+^ vaccine reduced total cholesterol, LDL-C, and VLDL-C by up to 44.7%, 51.7%, and 19.2%, respectively, after the fourth vaccination booster, compared with the control group at week 8. Long-term studies of vaccinated hypercholesterolemic mice revealed that the L-IFPTA^+^ vaccine was able to induce a long-lasting humoral immune response against PCSK9 peptide, which was paralleled by a significant decrease of LDL-C by up to 42% over 16 weeks post-prime immunization compared to control. Splenocytes isolated from the vaccinated group showed increased IL-10-producing cells and decreased IFN-γ-producing cells when compared with control and naive mice, suggesting the immune safety of the vaccine.

**Conclusions:**

L-IFPTA^+^ vaccine could generate long-lasting, functional, and safe PCSK9-specific antibodies in C57BL/6 mice with severe atherosclerosis, which was accompanied by long-term therapeutic effect against hypercholesterolemia and atherosclerosis.

## Background

Atherosclerotic cardiovascular disease (ASCVD) is the main cause of morbidity and mortality worldwide. ASCVD slowly progresses over the lifetime and becomes clinically manifest after several decades [1]. Active vaccination through the administration of immunogenic antigens to elicit an individual’s immune system to generate a humoral immune response is a highly effective and long-lasting method that could be used for preventing or treating ASCVD, though clinical evidence is lacking at the moment. However, passive immunotherapies based on monoclonal antibodies (mAbs) have improved the treatment of many chronic diseases including ASCVD [2, 3].

Low-density lipoprotein cholesterol (LDL-C) exerts a causal effect on atherosclerosis initiation and progression [1]. Various LDL-lowering methods, particularly statin therapy, that decrease LDL-C through upregulation of the LDL receptor (LDLR) have been revealed to decrease the risk of ASCVD events proportional to the absolute reduction of LDL-C in numerous randomized trials [1]. Although statin therapy is the most commonly used approach to treat hypercholesterolemia, there might be a relatively large number of patients that are statin-resistant or statin-intolerant and unable to achieve optimal LDL-C levels despite intensive statin therapy [4, 5].

Proprotein convertase subtilisin/kexin type 9 (PCSK9) is an important LDLR regulator that is involved in the progression of autosomal dominant hypercholesterolemia (ADH) [6]. Based on the recent mechanistic, genetic, and clinical evidence, PCSK9 has been identified as an important regulator of plasma LDL-C and as a therapeutic target [7–9]. PCSK9 mAbs, in combination with statins and/or ezetimibe, effectively decrease LDL-C by up to 50–60% and have now been shown to decrease the risk of ASCVD events proportional to the absolute reduction in LDL-C in two large-scale outcomes trials [3, 10, 11]. However, due to their relatively short in vivo half-life leading to frequent administration and high-cost, long-term clinical application of mAbs can be undesirable for many patients. Of note, growing evidence is emerging to suggest that the causal relationship of LDL-C with the risk of atherosclerosis is influenced by both the absolute magnitude and the total time of exposure to LDL-C [1]. Importantly, as arisen from Mendelian randomization studies, long-term exposure to LDL-lowering therapy beginning in early adulthood is correlated with up to a three-fold higher reduction in the risk of ASCVD events per unit change in LDL-C when compared with short-term therapy with a statin primed later in life [12]. Thus, initiation of LDL-lowering therapy earlier in life may inhibit or slow the development of atherosclerotic lesions and therefore could be an effective strategy to decrease the lifetime risk of ASCVD events. For this reason, the shift to primeval and long-lasting prevention of the atherosclerotic lesion formation by reducing LDL-C earlier in life will need new approaches that are safe, specific, well-tolerated, and easy to use [13].

Therefore, an active vaccination targeted against circulating PCSK9 if given in early adulthood before developing mature atherosclerotic lesions has the potential to decrease lifetime exposure to plasma LDL-C and may consequently result in potentially strong reductions in the lifetime risk of ASCVD events. A number of PCSK9-based vaccine strategies for reducing LDL-C are under investigation in preclinical or clinical phases [14–17]. Different approaches have in common that peptide vaccines can be chemically synthesized or produced by recombinant strategies. Hence, anti-PCSK9 vaccines can be produced at a much lower cost compared with the anti-PCSK9 antibodies that are required to be administrated regularly.

However, the peptide antigens generally show low immunogenicity and, therefore, need to be improved. Adjuvant systems are the effective approach commonly used in vaccine development for enhancing the immunogenicity of the peptide antigens. The peptide-based anti-PCSK9 vaccines prepared by other research groups contained adjuvants such as keyhole limpet hemocyanin (KLH) [18], DNA [14], and virus-like particles [16], which strongly increased the immunogenicity, though there are some concerns regarding their safety and efficiency in human.

An appropriate strategy to elicit strong antibody responses against self-antigens is to display them in a repetitive and highly dense format [19, 20]. Liposome nanoparticles are safe bilayer spherical vesicles that have been frequently used as adjuvant delivery systems in vaccine formulations. They are a feasible carrier for displaying antigens in peptide-based vaccines [21]. Our previous study showed that negatively charged nanoliposomes as an adjuvant delivery system could efficiently provoke a humoral immune response against exposed antigens. It was found that vaccines containing PCSK9 peptide exposed on the nanoliposome surface could induce long-term, strong, safe, and specific antibodies against PCSK9 in BALB/c mice [22]. Thus, the present study was aimed to evaluate the long-term therapeutic effect of nanoliposome-displayed PCSK9 as an alternative peptide-based vaccine for the treatment of hypercholesterolemia and atherosclerosis in C57BL/6 mice.

## Methods

### Construction and characterization of liposomal vaccine

The present studied liposomal vaccine engaging a peptide construct with immunogenic properties displayed on the surface of nanoliposome particles was fabricated as described in the following sections and as detailed in our previous report [22].

#### Preparation of liposome nanoparticles

To prepare nanoliposomes, cholesterol (Chol), 1,2-dimyristoyl-sn-glycero-3-phosphorylcholine (*DMPC*), and 1,2-dimyristoyl-sn-glycero-3-phosphorylglycerol (*DMPG*) (Avanti Polar Lipid; Alabaster, USA) lipids were dissolved in chloroform at the molar ratios of 15:10:75, respectively. Lipid solution was dried to a thin lipid film under reduced pressure using rotary evaporation (Heidolph, Germany). The prepared lipid film was then freeze-dried (VD-800F, Taitech, Japan) overnight to completely remove the solvent. Subsequently, the dried lipids were hydrated with 10 mM HEPES buffer (pH 7.2) containing 5% dextrose, and vortexed and bath-sonicated to disperse completely in the buffer. To obtain small unilamellar vesicles (SUVs) with a uniform size of 100–200 nm, the multilamellar vesicles (MLVs) were sequentially extruded using a mini extruder (Avestin, Canada) with polycarbonate membranes of 600, 400, 200, and 100 nm pore size, respectively. Physical properties of the prepared nanoliposomes, including particle size (diameter, nm), polydispersity index (PDI), and surface charge of the nanoliposomal formulation, were determined using dynamic light scattering (DLS) technique on a Zetasizer (Nano-ZS, Malvern, UK) at the room temperature (RT). The morphology and structure of the manufactured nanoliposomes were also visualized using a Philips CM10 transmission electron microscope (TEM).

#### Assembling of immunogenic peptide

A PCSK9 epitope, inspired the peptide sequence from the AFFiRiS group [18], was selected to induce antibodies targeting plasma circulating PCSK9. The selected peptide provides a B cell epitope, originally designed using *AFFITOME® technology* [23], that mimics an N-terminal sequence of the native PCSK9 bound to LDLR, and thereby can induce anti-PCSK9 antibodies inhibiting PCSK9/LDLR interaction. Furthermore, to provide a T helper cell epitope increasing the response of CD4^+^ T cells, a tetanus toxin peptide [24] was embedded in the PCSK9 fragment using a 2-lysine-spacer sequence. The peptide construct embracing PCSK9 and tetanus epitopes called immunogenic fused PCSK9-tetanus (IFPT) peptide (Additional file 1: Table S1) with a purity grade of > 95% was synthesized by ChinaPeptides Co., Ltd. (Shanghai, China).

#### Manufacturing of nanoliposomal IFPT vaccine

To expose IFPT peptide on the surface of the prepared liposome nanoparticles, it was linked to DSPE-PEG-Mal (1,2-distearoyl-*sn*-glycero-3-phosphoethanolamine-*N*-[maleimide (PEG)-2000])*lipid* (Lipoid GmbH, Germany) (Additional file 1: Figure S1). To approve the linkage of DSPE-PEG-Mal and IFPT peptide, a thin-layer chromatography (TLC) method was employed. Afterward, the DSPE-PEG-IFPT micelles were prepared using the solvent evaporation method followed by hydration. To quantify the peptide content of the micelles, high-performance liquid chromatography (HPLC) analysis (Knauer; Berlin, Germany) using an isocratic mobile phase of (0.1% TFA in water)/(0.1% TFA in acetonitrile) at gradient ratios of 55/45 to 45/55 in 10 min, at a flow rate of 1 mL min^−1^, was operated. The efficiency of the linkage in the assembled DSPE-PEG-IFPT micelles was estimated by subtracting the HPLC-measured amount of free peptide within the micelles from the amount of the initially used IFPT peptide. The IFPT peptide was displayed on the surface of nanoliposome particles using the post-insertion method (Additional file 1: Figure S2), in which the prepared DSPE-PEG-IFPT micelles (100 μg, based on the linked peptide) and nanoliposome formulation (1 mL) were mixed and then gently shaken at 45 °C for 3 h. Morphological and physical properties of the prepared liposomal IFPT (L-IFPT) were determined using DLS and TEM, respectively, as employed for free nanoliposomes. To finalize the vaccine package, the prepared L-IFPT formulation was adsorbed to 0.4% alum adjuvant (Sigma-Aldrich) at a 1:1 (v/v) ratio and stored at 4 °C under argon.

### Animal study

Twenty 6–8-week-old male C57BL/6 mice (18 ± 4 g) were purchased from the Laboratory Animal Research Center of Pasteur Institute of Tehran, Iran. All animal handling procedures were carried out in strict accordance with the Animal Welfare guidelines approved by the Institutional Ethics Committee and Research Advisory Committee of the Mashhad University of Medical Sciences, Mashhad, Iran. The animals were housed in an air-conditioned room at a constant temperature of 22 ± 2 °C with 12:12-h light/dark cycle and fed a standard rodent diet and water ad libitum. At the end of the study, all animals were euthanized by intravenous injection (30 mg/kg) of thiopental sodium [25, 26].

#### Induction of atherosclerotic lesion

Poloxamer 407 (P-407) is a non-ionic surfactant that through modulating activity of several key enzymes implicated in lipid metabolism and transport, including inhibition of cholesterol 7α-hydroxylase (C7αH), lipoprotein lipase (LPL), and hepatic lipase (HL) as well as inducing activity of cholesteryl-ester-transfer-protein (CETP) and lecithin cholesterol acyltransferase (LCAT), can induce hyperlipidemia in rodents [27, 28]. P-407 is also reported to decrease protein expression of liver LDLR [29, 30] and, along with the simultaneous ingestion of atherogenic diet, promote atherosclerosis lesions in either sex of C57BL/6 mice, similar to those formed in humans [31]. Here, to make a mouse model of atherosclerosis, 20 male 6–8-week-old C57BL/6 mice, weighting 18–23 g, were used. In order to induce atherosclerotic lesion, the animals fed with an atherogenic diet (containing 20% fat, 1.5% cholesterol, and 0.5% cholic acid) were simultaneously treated every third day with an intraperitoneal injection of P-407 (0.5 g kg^−1^) for a time period of 16 weeks [31]. After 16 weeks, to confirm atherosclerotic lesion development, the aortic arc region was isolated from 5 randomly selected mice.

#### Vaccination plan

To determine the therapeutic effect of the prepared vaccine on hypercholesterolemia and atherosclerosis development, the study design was planned in such a way that, initially, mouse model of atherosclerosis (described above) was developed and after that immunization schedule was primed (Additional file 1: Figure S3). Twenty male C57BL/6 mouse model of atherosclerosis were randomly and equally divided into two groups, including vaccine group and free nanoliposome (negative control) group. The vaccine group was immunized four times subcutaneously with L-IFPTA^+^ vaccine (200 μL in both the right and left flanks) in bi-weekly intervals [a modified method taken from Galabova’s study [18]]. Simultaneously, the negative control group received free nanoliposomes (200 μL) via the subcutaneous route, four times in bi-weekly intervals.

The time point at which the first inoculation was performed in order to induce anti-PCSK9 antibody refers to week 0 (W0) when it was simultaneous with 14 weeks of atherogenic regimen. Two weeks after the first immunization (W2), mice were put on a chow diet. Three more boosters were then carried out at W2, W4, and W6. To evaluate anti-PCSK9 antibody titers and lipid profile, the blood was withdrawn 2 weeks after each vaccination and at the pre-defined time points during 16 weeks after the first vaccination (Additional file 1: Figure S3).

### Measuring the plasma level of anti-PCSK9 peptide antibody

Plasma samples isolated from vaccinated hypercholesterolemic and the negative control mice were assayed by the ELISA method to measure the titers of the induced antibodies against PCSK9 peptide. Briefly, a 96-well Nunc-MaxiSorp plate was coated with PCSK9 peptide solution at the concentration of 5 μg/mL in 0.1 M NaHCO_3_ buffer (pH 9.2–9.4), through an overnight incubation at 37 °C. Afterward, a blocking buffer (1× PBS, 1% BSA) was incubated on the coated plate for 1 h at 37 °C to bock free binding sites. Diluted plasma (1:400 in 1× PBS/0.1% BSA/0.05% Tween-20) was added, serially diluted 1:4, and incubated for 1 h at 37 °C. Each ELISA plate contained a standard antibody as the internal control. For the detection, biotinylated anti-mouse IgG (H+L) (Sigma-Aldrich; 1:1000) in 1× PBS/0.1% BSA/0.1% Tween-20 was incubated for 1 h at 37 °C. As the next step, horseradish peroxidase coupled to streptavidin (Sigma-Aldrich) was added (30 min, 37 °C) followed by the addition of the substrate TMB (Sigma-Aldrich) (15 min, RT). The optical density (OD) at 450 nm was measured with a microwell plate reader (BioTek, Synergy 2 plate reader, VT, USA), and the titers were defined as the dilution factor referring to 50% of the maximal optical density (OD_max_/2). The mean titers ± SEM of all animals per group are presented.

### Plasma PCSK9 quantification

Plasma PCSK9 levels of hypercholesterolemic vaccinated and the negative control mice were quantified by CircuLex mouse PCSK9 ELISA (CircuLexTM, Cy-8078, MBL, Woburn, MA) according to the manufacturer’s instructions. Briefly, 100 μL of the diluted 1:100 plasma samples was incubated on a 96-well microplate for 1 h at RT. An HRP-conjugated anti-PCSK9 antibody was incubated for 1 h followed by the substrate reagent and stop solution, all at RT. OD was measured at 450 nm with the microwell plate reader. Finally, to determine the PCSK9 level, a standard curve provided by the supplier was defined.

### Evaluation of mouse PCSK9 targeting

To assess targeting of mouse PCSK9 by vaccine-generated antibodies, the interaction of plasma antibodies with PCSK9 was determined. To this, a modified method of CircuLex mouse PCSK9 ELISA kit was employed. In brief, to detect PCSK9-bound plasma antibodies, HRP-conjugated anti-mouse IgG (H+L) (Sigma Aldrich; dilution 1:5000, incubated for 1 h at RT), instead of HRP-conjugated anti-PCSK9 antibody, was used. Subsequently, PCSK9-targeting plasma antibody of vaccinated mice was indicated using detected OD at 450 nm.

### Inhibitory effect of the induced antibodies on PCSK9/LDLR interaction in vitro

The ability of vaccine-generated antibodies for inhibition of the PCSK9/LDLR interaction in vitro was evaluated using PCSK9-LDLR in vitro binding assay kit (CircuLex™, Cy-8150, MBL, Woburn, MA). The principle of the assay is based on the binding between recombinant His-tagged PCSK9 and recombinant epidermal growth factor-like repeat (EGF-A) domain of LDLR, which contains a binding site for PCSK9. A biotinylated anti-His tag monoclonal antibody (supplemented with the company) specifically targets recombinant His-tagged PCSK9 that has been trapped with recombinant EGF-A domain coated on the microplate surface. Therefore, when evaluating a candidate PCSK9 inhibitor, if it can target the EGF-A binding domain of PCSK9, it will decrease the reaction of a biotinylated anti-His tag monoclonal antibody with His-tagged PCSK9 and consequently decrease subsequent detected OD. Briefly, 100 μL/well of the plasma samples of vaccinated mice or vehicle control was added to a 96-well microplate pre-coated with a recombinant LDLR-EGF-A domain. Immediately after that, the reaction was initiated by adding a “His-tagged PCSK9” solution incubated for 2 h followed by adding a biotinylated anti-His tag monoclonal antibody for 1 h at RT. Then, HRP-conjugated streptavidin was coated for 1 h at RT followed by the substrate reagent and stop solution. In this method, the higher amount of PCSK9-LDLR interaction is associated with higher ELISA OD, in which at the presence of anti-PCSK9 antibody, this interaction is inhibited and consequently ELISA OD is decreased. A dose-response curve with appropriate serial dilutions of “His-tagged PCSK9 wild-type” solution was drawn to measure accurate inhibition percentage of test samples.

### Plasma lipid quantification

Peripheral blood was collected, and total cholesterol (TC), direct LDL-C, very low-density lipoprotein cholesterol (VLDL-C), and triglyceride (TG) were measured using the Biosystems kits (Biosystems S.A., Barcelona, Spain).

### Histological assessment of atherosclerosis

At the end of the study, mice were euthanized and atherosclerotic lesion size and severity were assessed in the aortic arc area. Briefly, the aortic arc identified by the appearance of aortic valve leaflets was cut and immersion-fixed in 10% buffered formalin. The formalin-preserved tissue was gradually dehydrated, embedded in paraffin, and serially cut into sections with 5 μm thickness and intervals of 50 μm. Then, the slides were de-paraffinized in p-xylene and rehydrated in ratios of ethanol (100, 80, 70, and 50%) and rinsed in water. To stain the histopathology slides, hematoxylin and eosin (H&E) staining was used. Briefly, slides were stained in hematoxylin for 5 min and rinsed with water. Afterward, the slides were counterstained in eosin and mounted in distyrene, tricresyl phosphate, and xylene (DPX). For the assessment of atherosclerotic lesion thickness and severity, the lesions were classified into an arbitrary scale of 1–4 [32]: *trace*, minimal thickening of subintima with little injury to arterial endothelium (early fatty streak); *grade 1*, plaque containing foam cells less than half as thick as the media with some form of endothelial dysfunction (regular fatty streak); *grade 2*, plaque at least half as thick as the media with accumulation of intracellular lipid, macrophages, and smooth muscle cells (mild plaque); *grade 3*, plaque as thick as the media with an abundance of macrophages, smooth muscle cells, and connective tissue (moderate plaque); and *grade 4*, plaque thicker than the media with evidence of large extracellular intimal lipid core, foam cells, and calcification in the lipid core (severe plaque). The lesions were checked out using light microscopy (Olympus BX 51 microscope) supplied with a digital camera under × 400 magnifications. The lesion area was analyzed with ImageJ software [33].

### Western blot analysis of liver LDLR

To evaluate the protein expression of mouse liver LDLR, western blot analysis and immunohistochemical staining were performed. Liver crude protein was extracted using RIPA lysis buffer 500 μL per mg tissue (Sigma-Aldrich) with sodium orthovanadate, phenylmethylsulfonyl fluoride, and proteinase inhibitors. SDS-PAGE 10% gel was loaded with 50 μg protein per lane. Blotted proteins were developed using an HRP-conjugated anti-LDLR goat IgG (R and D Systems, Minneapolis, MI) diluted in primary antibody diluent buffer. HRP-conjugated anti-tubulin (Sigma, St. Louis, MO) mouse mAb was used to normalize data. Bands were visualized by Gel Documentation System (Bio-Rad) and quantified by ImageJ software.

### Immunohistochemical staining for liver LDLR

Mouse liver sections were fixed in 10% buffered formalin and embedded in paraffin. Sections of 10 μL were obtained using a microtome, cleared in xylol, and rehydrated. The unmasking procedure was performed by incubating the samples in an antigen retrieval solution (EDTA buffer; pH 9.0) at 99 °C for 40 min. After rinsing in PBS, the sections were incubated with blocking solution (15 μL goat serum in 1 mL PBS) for 30 min at RT and then without an additional rinse, immediately incubated with rabbit monoclonal anti-LDLR antibody (Abcam Inc., Cambridge, UK) at the dilution of 1:500 for 1 h at RT. The samples were then rinsed in PBS and incubated with goat anti-rabbit HRP-conjugated IgG antibody (Sigma-Aldrich Inc., St. Louis, MO) at the dilution of 1:200 for additional 60 min. To counterstain the samples, the nuclei were stained with hematoxylin. The sections were dehydrated and mounted with Entellan (Merck KGaA, Darmstadt, Germany).

### Evaluation of inflammatory response using ELISpot method

At the end of the study, the vaccinated hypercholesterolemic mice, non-vaccinated hypercholesterolemic mice, and naive mice (five animals per group) were sacrificed and their splenocytes were aseptically isolated, homogenized, and then passed through a 70-μm cell strainer (BD Falcon). The red blood cells (RBCs) were lysed using ACK buffer (0.15 M NH4Cl, 1.0 M KHCO3, 0.1 mM Na2EDTA), and the RBC-depleted splenocytes were counted using trypan blue (Gibco). INF-γ and IL-10 cytokines were assayed using the Mouse INF-γ and IL-10 ELISpot Kit (Mabtech), respectively, according to the manufacturer’s protocol. Briefly, 100 μL/well of either 15 μg/mL anti-INF-γ or anti-IL-10 antibody solution (diluted in sterile PBS pH 7.4) was coated on 96-well PVDF plates (Millipore Corp.) through an overnight incubation at 4 °C. To block non-specific binding, 200 μL/well blocking buffer containing RPMI medium (Gibco) supplemented with 10% fetal calf serum (FCS) (Gibco) was incubated on the coated plates for 30 min at RT. The blocked plates were seeded with the isolated splenocytes (5 × 10^5^ cells per well) and re-stimulated either with 20 μg/mL phytohemagglutinin (PHA) (Sigma-Aldrich) or supplemented RPMI medium and incubated for 24 h at 37 °C. Eventually, spot-forming cells (SFC) were detected according to the manufacturer’s guidelines, and the amount of INF-γ- and IL-10-producing cells was quantified by counting the number of spots per well using Kodak 1D image analysis software (Version3.5, Eastman Kodak, Rochester, NY). Values were expressed as the number (median-interquartile range) of anti-INF-γ and/or anti-IL-10 SFC per 10^6^ cells.

### Statistical analysis

To determine the significance of the difference among the groups, unpaired two-tailed Student’s *t* test and one-way ANOVA followed by Tukey’s post hoc test were employed (GraphPad Prism software, version 7, San Diego, CA). Data with *p* < 0.05 were considered to be statistically significant.

## Results

### Characterization of nanoliposomal formulations

Physical properties of the free nanoliposome formulations, including size, PDI, and zeta potential, are shown in Additional file 1: Table S2. The free nanoliposomes and the IFPT-linked nanoliposomes exhibited a size range from 137 to 165 nm in diameter, in which PDI was less than 0.02, showing homogeneity of particles (Additional file 1: Figure S4). Zeta potential analysis also revealed a negative charge on the surface of nanoparticles (Additional file 1: Figure S5). The nanoliposomal vesicles were visualized by transmission electron microscopy indicating unilamellar vesicles with the lamellae of the vesicles evenly spaced to the core as shown in Additional file 1: Figure S6.

### TLC and HPLC analysis of DSPE-PEG-IFPT micelles

Based on the disappearing of DSPE-PEG-Mal spot (lipid spot) on the TLC plate, conjugation of DSPE-PEG-Mal linker and the IFPT peptide was verified after 48 h reaction (Additional file 1: Figure S7). Afterward, DSPE-PEG-IFPT micelles were made, and the efficiency of conjugation was measured using HPLC analysis, indirectly, by quantification of the free peptide content of the micelle sample. HPLC analysis indicated that 96% of the initially added IFPT peptides were conjugated to the DSPE-PEG-Mal linker (Additional file 1: Figure S8).

### Liposomal vaccine induces high antibody titers in hypercholesterolemic C57BL/6 mice

L-IFPTA^+^ vaccine significantly and highly elicited IgG antibody response against PCSK9 peptide in hypercholesterolemic mice upon four immunizations. The ELISA analysis revealed that anti-PCSK9 antibody titer was 1:42500 ± 3200 after the last immunization (Fig. 1a). The long-term analysis revealed that anti-PCSK9 antibody titers reached their peak levels at week 8 and remained constant up to week 12 and then showed the reduced trend. To sum up, the results indicate an efficient adjuvant activity of nanoliposomes to induce humoral immunoresponse against peptide antigen.

**Fig. 1:** Efficacy of L-IFPTA^+^ vaccine against in hypercholesterolemic C57BL/6 mice, 2 weeks after the last vaccination. **a** Antibody titers (OD_max_/2) against PCSK9 in vaccinated hypercholesterolemic C57BL/6 mice. **b** Plasma concentration of PCSK9 in the vaccinated and control groups was 116.8 ± 8 ng/mL and 281.5 ± 5.2 ng/mL, respectively. **c** Direct detection of antibodies bound to plasma PCSK9 in the blood samples from vaccinated and control mice. Elevated OD450 is indicative of vaccine-induced anti-PCSK9 antibodies directly binding to PCSK9. **d** In vitro PCSK9/LDLR binding assay. Vaccine-induced antibodies inhibited PCSK9/LDLR interaction. The plasma sample of the L-IFPTA^+^ vaccine group could decrease PCSK9 binding to LDLR by 44.8%, when compared with the plasma sample of the control group. Bars show mean values; error bars show ± SD (*n* = 3 replicates of the pooled samples of 10 mice per group). Significance compared to control values was analyzed by unpaired two-tailed Student’s *t* test

### Vaccine-generated anti-PCSK9 antibodies target plasma PCSK9

To evaluate specific targeting of vaccine-induced anti-PCSK9 antibodies in vivo, plasma levels of PCSK9 in vaccinated mice were evaluated. Vaccine-induced anti-PCSK9 antibody was found to specifically target plasma PCSK9 in hypercholesterolemic C57BL/6 mice. Hence, plasma levels of PCSK9 in the L-IFPTA^+^ vaccine and control groups were 116.8 ± 8 and 281.5 ± 5.2 ng/mL, respectively (Fig. 1b). Compared with the control mice, plasma levels of PCSK9 were significantly decreased by 58.5% (− 164.7 ± 9.6 ng/mL, *p =* 0.0001) in vaccinated mice. For further evidence of specific targeting, PCSK9 inhibition was evaluated using ELISA-based assay to detect vaccine-generated antibodies directly bound to plasma PCSK9. For this aim, plasma PCSK9 from vaccinated and control mice was captured onto murine anti-PCSK9 antibody-coated ELISA plates, and vaccine-generated PCSK9-bound antibodies were detected using an anti-mouse IgG antibody. As shown in Fig. 1c, the significantly higher OD450 signal in the plasma of mice vaccinated with L-IFPTA^+^ vaccine confirmed a direct binding of vaccine-generated anti-PCSK9 antibodies to the target protein (PCSK9). To sum up, L-IFPTA^+^ vaccine induces specific antibodies that directly target and bind mouse PCSK9 in the bloodstream.

### Vaccine-generated anti-PCSK9 antibodies inhibit in vitro PCSK9/LDLR interaction

As detected by PCSK9/LDLR in vitro binding assay kit, vaccine-induced anti-PCSK9 antibodies from hypercholesterolemic C57BL/6 mice could efficiently inhibit PCSK9/LDLR interaction in vitro. The plasma sample of the L-IFPTA^+^ vaccine group could significantly decrease PCSK9 binding to LDLR by 44.8%, when compared with the plasma sample of the control group (Fig. 1d). The results showed that induced antibodies could inhibit PCSK9 function through direct targeting of the EGF-A binding domain and, thereby, inhibiting PCSK9-mediated LDLR degradation.

### Lipid-lowering effect of liposomal vaccine in hypercholesterolemic C57BL/6 mice

To evaluate the therapeutic effect of L-IFPTA^+^, C57BL/6 mice were placed on an atherogenic regimen for 16 weeks, and 2 weeks before the end of the regimen period (week 14), mice were immunized, in which the prime vaccination refers to week 0 (Additional file 1: Figure S3). The functional therapeutic effect of L-IFPTA^+^ vaccine against PCSK9 was assessed by measuring the cholesterol levels in the vaccinated hypercholesterolemic C57BL/6 mice before and after immunization (Fig. 2). L-IFPTA^+^ vaccine managed cholesterol levels in hypercholesterolemic C57BL/6 mice upon immunization. Two weeks after the last vaccination (week 8) relative to pre-vaccination (week 0), the L-IFPTA^+^ vaccine could significantly decrease plasma levels of TC (Fig. 2a), LDL-C (Fig. 2b), and VLDL-C (Fig. 2c) by 750 ± 43.8 mg/dL, 132.4 ± 6 mg/dL, and 242 ± 10.5 mg/dL, respectively, while at the same time period in the negative control group, TC, LDL-C, and VLDL-C were decreased by 518.6 ± 44 mg/dL, 87.3 ± 5.8 mg/dL, and 222.7 ± 11 mg/dL, respectively. There was no significant difference in plasma TG levels between the vaccinated and control groups (Fig. 2d). Compared with the negative control group, the plasma levels of TC, LDL-C, and VLDL-C were decreased by 44.7%, 51.7%, and 19.2%, respectively, in the hypercholesterolemic C57BL/6 mice after the fourth vaccination.

**Fig. 2:** Quantification of plasma lipids in hypercholesterolemic mice, in pre-vaccination (week 0) and after four vaccinations (post-vaccination; week 8) with L-IFPTA^+^ vaccine. Mean and SEM are demonstrated for **a** total cholesterol, **b** LDL-C, **c** VLDL-C, and **d** triglyceride. Negative control involves hypercholesterolemic mice received free liposomes. Each data point symbolizes an individual mouse; lines represent means for each group. Significance values were calculated by comparison with control values using a two-tailed Student’s *t* test. LDL-C, low-density lipoprotein cholesterol; VLDL-C, very low-density lipoprotein cholesterol; ns, not significant

### LDL-C levels inversely correlate with anti-PCSK9 antibody titers in vaccinated mice

Analysis of the anti-PCSK9 antibody levels reported above shows that the average antibody titers from the hypercholesterolemic vaccinated mice were significantly higher than the mean titers measured on the negative control group. Consistently, the average level of circulating LDL-C in hypercholesterolemic vaccinated mice was lower than that measured in the negative control group. As illustrated in Fig. 3, there was a significant inverse correlation between LDL-C levels and anti-PCSK9 antibodies titers, in which anti-PCSK9 antibodies and LDL-C levels being respectively at the highest and lowest levels in the hypercholesterolemic vaccinated mice. Thus, the nanoliposomal anti-PCSK9 L-IFPTA^+^ vaccine provokes high anti-PCSK9 titers that directly associate with the reduction in plasma LDL-C levels.

**Fig. 3:** Correlation between plasma levels of LDL-C and anti-PCSK9 antibody titers in immunized mice. Correlation plot of circulating LDL-C levels with anti-PCSK9 antibody titers evaluated throughout 8 weeks post-prime immunization. A significant anti-correlation was identified among LDL-C levels and the anti-PCSK9 antibody titers in hypercholesterolemic C57BL/6 mice upon four vaccinations (*r* = − 0.99, *p* = 0.0009)

### Long-term therapeutic efficacy of liposomal vaccine in hypercholesterolemic mice

To understand the persistence of the induced anti-PCSK9 antibody and correlated cholesterol-lowering effect, a long-term study was undertaken on hypercholesterolemic vaccinated mice. Antibody titer analyses over 16 weeks post-prime immunization revealed that L-IFPTA^+^ vaccine was able to stimulate a long-lasting humoral immune response against PCSK9 peptide (Fig. 4a), which was paralleled by a significant decrease of LDL-C by up to 127.7 ± 7.4 mg/dL (Fig. 4b). Compared with the negative control group, plasma levels of LDL-C were decreased by 42% in the hypercholesterolemic C57BL/6 mice over 16 weeks post-prime immunization.

**Fig. 4:** Long-term therapeutic efficacy of L-IFPTA^+^ vaccine in hypercholesterolemic C57BL/6 mice. **a** Evaluation of anti-PCSK9 antibody titers (OD_max_/2) over 16 weeks post-prime vaccination, generated upon four immunizations in a bi-weekly interval (signed by arrows). Values are means ± SD, *n* = 7 mice/group. **b** Measurement of LDL-C levels over the same time period as **a**. Values are means; error bars represent SDs (*n* = 7 mice/group). To compare the L-IFPTA^+^ vaccine and control groups, two-way ANOVA test was used, followed by Bonferroni multiple comparisons test, at the indicated time points

### The liposomal vaccine increases the liver LDLR in hypercholesterolemic mice

To determine the effect of anti-PCSK9 antibody titers on the levels and cellular distribution of the liver LDLR protein in vaccinated hypercholesterolemic mice, western blot analysis and IHC staining were carried out (Fig. 5). The liver LDLR protein was visualized and quantified by western blotting with an anti-LDLR antibody (Fig. 5a). The level of hepatic LDLR protein in hypercholesterolemic mice vaccinated with L-IFPTA^+^ vaccine was 3.75 ± 0.55-fold higher than in the negative control group (Fig. 5b). IHC analyses of the same liver samples exhibited a comparable staining of the cell membrane and cytoplasm (Fig. 5c), whereas samples from vaccinated mice exhibited a significant enhanced staining at the cell membrane (Fig. 5d). Therefore, our analysis shows an increase in the cell surface levels of liver LDLR in immunized versus control mice.

**Fig. 5:** Expression (**a**, **b**) and cellular distribution (**c**, **d**) of LDLR in the livers of immunized hypercholesterolemic mice. Liver extracts were separated by SDS-PAGE and blotted onto a nitro-cellulose filter. Following incubation with HRP-conjugated anti-LDLR or anti-β actin antibody, the bands corresponding to LDLR or β-actin proteins were measured by ImageJ software. The LDLR bands were normalized on the corresponding β-actin band (**a**). Compared to the control group, the protein expression of LDLR in the liver was significantly increased in the vaccine group. Data are expressed as means ± SEM (*n* = 7 per group). Differences at *p* values less than 0.05 were considered to be statistically significant (**b**). The cellular distribution of LDLR in immunized mice (**c**, **d**). Immunohistochemistry analysis was carried out on the liver samples isolated from the control (**c**) or vaccinated (**d**) mice using rabbit anti-LDLR antibodies detected by anti-rabbit IgG HRP-conjugated antibodies

### Liposomal vaccine decreases the size and severity of atherosclerotic lesion in the aorta

To assay the impact of L-IFPTA^+^ vaccine on atherosclerotic lesion progression in mouse model of atherosclerosis, the aortic arc was isolated and the lesion size, intima to media thickness, (IMT), and lesion grade were determined using H&E staining (Fig. 6). Representative images of aortic arch lesions of IFPTA^+^ and control mice are depicted in Fig. 6a. L-IFPTA^+^ vaccine could significantly decrease the lesion size (39.13%, *p =* 0.016) and IMT (46%, *p* = 0.003) compared with the negative control (Fig. 6b, c). The lesion severity was categorized according to an arbitrary scale of 1–4 grade [32]. Although the relative amount of mild lesions (grade II) was similarly distributed between L-IFPTA^+^ (29%) and control (43%) mice, the more severe lesions (grade III and IV) were only observed in 57% of control mice, while 71.5% of IFPTA^+^ mice showed grade I and 0 lesions (Fig. 6d). A strong positive correlation between the atherosclerotic lesion size and plasma LDL-C (*r* = 0.75, *p* = 0.001) as well as plasma PCSK9 levels (*r* = 0.61, *p* = 0.004) was observed.

**Fig. 6:** Inhibitory effect of LIFPT-A^+^ vaccine on the development of atherosclerotic lesion in the aortic arc area of C57BL/I mouse model of diet-induced atherosclerosis. Sixteen weeks after, the prime vaccination of mice on severe atherogenic diet lesion development was determined using hematoxylin and eosin (H&E) staining. **a** Representative views of H&E-stained grade I, II, and III lesions of the aortic arc. **b** Lesion size in vaccinated and control mice was 70.43 ± 14.56 μm and 115.4 ± 7.164 μm, respectively. Lesion size was found to be 39.13% (− 45 ± 16.22 μm, *p =* 0.016) lower in vaccinated mice than in control mice. Data are expressed as group means ± SD (*n* = 7 mice per group). Significance compared to control values was analyzed by unpaired two-tailed Student’s *t* test. **c** Intima to media thickness (IMT) in vaccinated and control mice was 0.4 ± 0.09 and 0.9 ± 0.05, respectively. IMT in the vaccine group was significantly decreased by 46% (0.42 ± 0.1, *p* = 0.003) compared with the control group. Data are expressed as group means ± SD (*n* = 7 mice per group). Significance compared to control values was analyzed by unpaired two-tailed Student’s *t* test. **d** Lesion grade in vaccinated and control mice was 1 [1, 2] and 3 [2, 3], respectively. Data are expressed as group medians [25% percentile–75% percentile] (*n* = 7 mice per group). Significance compared to control values was analyzed by Mann-Whitney *U* test

### Anti-inflammatory effect of liposomal vaccine in hypercholesterolemic C57BL/6 mice

As revealed by ELISpot analysis of splenic cells, therapeutic use of L-IFPTA^+^ vaccine was shown to be immunologically safe and enhanced anti-inflammatory response in hypercholesterolemic C57BL/6 mice. IFN-γ secretion was found to be increased in hypercholesterolemic mice by 2.32-fold, when compared with naive mice. L-IFPTA^+^ vaccine could inhibit IFN-γ production in hypercholesterolemic mice, in which levels of splenocyte-secreted IFN-γ in vaccinated hypercholesterolemic mice were 0.68-fold lower than those in the hypercholesterolemic mice (Fig. 7a, c). Levels of splenocyte-secreted IL-10 in vaccinated hypercholesterolemic mice were 2.1- and 2.41-fold higher than those in hypercholesterolemic and naive mice, respectively (Fig. 7b, d).

**Fig. 7:** Representative IFN-γ (**a**) and IL-10 (**b**) ELISPOT wells for the splenocytes isolated from various treatment groups. ELISpot analysis revealed that IFN-γ production by splenic cells isolated from vaccinated hypercholesterolemic mice was significantly decreased (**c**), while production of IL-10 was significantly increased (**d**), when compared with hypercholesterolemic mice. The isolated splenocytes were stimulated with PHA (as positive control) or medium. Data are presented as mean ± SD, 7 mice/group

## Discussion

mAb-based PCSK9 inhibitors can effectively lower high levels of LDL-C but their long-term clinical application necessitates frequent administration and high cost [34]. To subdue such limitation, active vaccination with long-lasting effects can be a safe alternative to passive immunotherapy of hypercholesterolemia [35, 36]. Active vaccination for PCSK9 inhibition has been investigated by different approaches. AFFiRiS group developed an AFFITOPE®-based anti-PCSK9 active vaccination approach using a PCSK9 peptide linked to KLH carrier, which reduced TC by 53% [18] and was associated with the reduction of size and severity of atherosclerotic lesion in vaccinated compared with control mice [17]. However, the results of phase I clinical trial revealed that the mentioned vaccine failed to mimic similar cholesterol-lowering effects in humans, as Bauer et al. reported a 13% reduction in cholesterol level of vaccinated subjects (Bauer et al., Communication at ESC Congress, 2018 Munich; unpublished data). This finding highlights the need for further development of the introduced PCSK9 vaccine. We are the first to exhibit anti-PCSK9 vaccine with a nanoliposomal adjuvant carrier (L-IFPTA^+^ vaccine) that exerted long-lasting lipid-lowering effects associated with anti-atherosclerotic effects in C57BL/6 mice receiving a severe atherogenic regimen.

In the present developed atherosclerosis model, a considerable reduction of plasma lipids occurred after stopping the atherogenic regimen. Therefore, to detect the net lipid-lowering effect of L-IFPTA^+^ vaccine, we included a negative control (free nanoliposomes or phosphate-buffered saline) without effects on plasma lipids as verified in a pilot study (Additional file 1: Figure S9). Hence, the reduced level of plasma lipids in the negative control group (Figs. 2 and 4) is due to the atherogenic diet discontinuation and not an effect of free nanoliposomes.

L-IFPTA^+^ vaccine-induced functional antibodies that specifically bound to circulating PCSK9 and inhibited its interaction with LDLR and thereby increased expression of LDLR on the surface of liver cells leading to significant reductions in TC and (V)LDL-C accompanied by a reduction in the atherosclerotic lesion size in the aortic arch of hypercholesterolemic mice. Upon four vaccinations with L-IFPTA^+^, plasma antibody titer reached peak levels, at which plasma levels of PCSK9 were significantly decreased by 58.5% in the vaccinated hypercholesterolemic mice compared with hypercholesterolemic mice received free nanoliposomes (negative control). When antibody titers reached maximum levels (week 8), plasma LDL-C was found to be at the minimum level, which was associated with a 51.7% decrease in the plasma levels of LDL-C. The long-term study showed that during 16 weeks after prime vaccination, plasma LDL-C levels significantly decreased in vaccinated hypercholesterolemic mice, when compared with the negative control. At the end of the study (week 16), L-IFPTA^+^ vaccine decreased LDL-C by 42% relative to the priming time point, showing a statistically significant negative correlation of antibody titers and LDL-C levels. Such a cholesterol-lowering effect was accompanied by the reduction of atherosclerotic lesion size (39.13%, *p =* 0.016) and severity (46%, *p* = 0.003) in the aortic arch of vaccinated hypercholesterolemic mice compared with the negative control. To the best of our knowledge, only one other group [17] reported that active vaccination against PCSK9 could reduce atherosclerosis development in APOE*3Leiden.CETP mice; however, we showed the atheroprotective effect of L-IFPTA^+^ in a different murine model of severe atherosclerosis. Regarding the intense induced hypercholesterolemia in our model, therapeutic effect of the present vaccine has the potential to be translated in patients with high levels of plasma cholesterol, suggesting its ideal benefit for future clinical use.

Furthermore, in another approach, Fattori et al. evaluated human recombinant PCSK9, together with a DNA oligonucleotide as an adjuvant, and reported ~ 40% reduction of LDL-C in mice [14]. Pan et al. developed a human PCSK9 vaccine in which PCSK9 peptides were displayed at high valency on the surface of a bacteriophage virus-like particle, leading to nearly 20% reduction of TC relative to controls [16]. However, it is questionable and unclear whether KLH [18], DNA [14], or virus-like particles [16] used in the aforementioned studies can be safe adjuvants for clinical practices. Hence, besides the higher cholesterol-lowering effect of L-IFPTA^+^ vaccine in comparison with other published PCSK9-targeting vaccines, it can rise important advantages of using safe adjuvant due to approved safety of liposome nanoparticles [37], and thereby provide a clear outlook for clinical use.

On the other hand, inflammation is found to play a key role in atherosclerosis progression and complications. There is growing evidence showing the pro-atherogenic role for IFN-γ-producing cells [38]. The pro-inflammatory IFN-γ cytokine could promote and exacerbate atherosclerosis via affecting the lipid accumulation and foam cell formation in the vascular wall and altering the cellular structure in the plaque, such as effects on SMC proliferation and macrophage activation [39]. In contrast, IL-10-producing cells could counteract IFN-γ production [40]. We showed that in the hypercholesterolemic control mice, IFN-γ-producing splenic cells were increased when compared with the naive mice on a chow diet. L-IFPTA^+^ vaccine was found to significantly decrease IFN-γ-producing splenic cells, compared with controls. It was also revealed that IL-10-producing splenic cells were significantly increased in vaccinated versus control mice. Our finding is in accordance with the report of AFFiRiS group that showed PCSK9-targeting vaccine could ameliorate systemic and vascular inflammation in the aorta in APOE*3Leiden.CETP mice [17]. The results can somewhat confirm the anti-inflammatory effect of L-IFPTA^+^ vaccine that could have contributed to the observed anti-atherosclerotic effects; however, assessment of inflammatory cell distribution in plaque is needed to definitely verify this effect. Furthermore, both IFN-γ and IL-10 cytokines are validated markers for systemic inflammation [41], and therefore, the present findings can provide the implications regarding the immunological safety of the L-IFPTA^+^ vaccine.

While the present study is the first to report the anti-atherosclerotic and cholesterol-lowering effect of a nanoliposome-based PCSK9 peptide vaccine, a number of limitations need to be acknowledged to guide future studies. These limitations include the need for the verification of results in additional models of atherosclerosis including the transgenic models of atherosclerosis such as *ldlr*-, *aopE*-, or *pcsk9*-deficient mice as well as in rhesus monkeys. Besides, long-term evaluations are also encouraged to provide more in-depth information on the impact of the introduced vaccine on the size, morphology, and composition of atherosclerotic plaques. The impossibility of evaluating the effect of L-IFPTA^+^ vaccine on the other atherogenic plasma factors, such as lipoprotein a (Lp(a)), due to the absence of the mentioned factor in rodents was another limitation that calls for future testing in specific genetically engineered models. Finally, to provide more information on the effect of L-IFPTA^+^ vaccine on atherosclerosis plaques, staining of plaque lipids using Oil Red O method could be useful.

## Conclusions

In conclusion, L-IFPTA^+^ vaccine could generate long-lasting, functional, and safe PCSK9-specific antibodies in a C57BL/6 mouse model of severe atherosclerosis. This results in a long-term therapeutic effect against hypercholesterolemia and atherosclerosis. Thus, the use of L-IFPTA^+^ vaccine could serve as a potential alternative to mAb-based therapies and could lead to a widely feasible vaccine-based tool for managing hypercholesterolemia and ASCVD. Nevertheless, further supportive evidence from the clinical setting is highly demanded.

## Supplementary information

**Additional file 1: Table S1**. Sequence of the immunogenic peptides used in the present study. **Table S2**. Physical properties of nanoliposomal formulations. **Figure S1**. Schematic view of linking between peptide and DSPE-PEG-Maleimide. **Figure S2**. Schematic view of post insertion process. **Figure S3**. Schematic diagram of study design. **Figure S4**. Representative graph indicated size and polydispersity index (PDI) of the empty nanoliposomes (**A)** and the IFPT linked-nanoliposomes (**B**). **Figure S5**. Representative graph indicated zeta potential of the empty nanoliposomes (**A)** and the IFPT linked-nanoliposomes (**B**). **Figure S6**. Transmission electron micrography of nanoliposome particles, showing unilamellarity, dispersity, and size of vesicles. **Figure S7**. Assessment of conjugation between DSPE-PEG-Mal and the IFPT peptide at the time zero and 48 h after starting the reaction. **Figure S8**. HPLC chromatogram of DSPE-PEG-IFPT micelles (A) and reference standard IFPT peptide. **Figure S9**. Plasma levels of total cholesterol (TC), low-density lipoprotein cholesterol (LDL-C), very low-density lipoprotein cholesterol (VLDL-C), and triglyceride (TG) during 4 weeks after discontinuing atherogenic regimen in the untreated hypercholesterolemic C57BL/6 mice, and those received free nanoliposomes or phosphate-buffered saline (PBS).

## Data Availability

Data are available from the corresponding authors upon reasonable request.

## Abbreviations

ASCVD: Atherosclerotic cardiovascular disease
ADH: Autosomal dominant hypercholesterolemia
EGF-A: Epidermal growth factor-like repeat
DLS: Dynamic light scattering
DMPC: 1,2-Dimyristoyl-sn-glycero-3-phosphorylcholine
DMPG: 1,2-Dimyristoyl-sn-glycero-3-phosphorylglycerol
HPLC: High-performance liquid chromatography
IFN-γ: Interferon-gamma
IFPT: Immunogenic fused PCSK9-tetanus
IL-10: Interleukin-10
IMT: Intima to media thickness
LDL-C: Low-density lipoprotein cholesterol
mAbs: Monoclonal antibodies
MLV: Multilamellar vesicles
OD: Optical density
PCSK9: Proprotein convertase subtilisin/kexin type 9
PDI: Polydispersity index
RIPA: Radioimmuneprecipitation assay
RT: Room temperature
SUV: Small unilamellar vesicles
TEM: Transmission electron microscope
